# RET receptor tyrosine kinase architecture, assemblies and activation

**DOI:** 10.1530/ERC-25-0322

**Published:** 2026-04-17

**Authors:** Mia Zol-Hanlon, Neil Q. McDonald

**Affiliations:** 1 Signalling and Structural Biology Laboratory, Francis Crick Institute, NW1 1AT, London, United Kingdom; 2 Institute of Structural and Molecular Biology, School of Natural Sciences, Birkbeck College, Malet Street, London, WC1E 7HX, United Kingdom

## Abstract

Among the 58 human receptor tyrosine kinases that are known, only the RET (REarrangement during Transfection) receptor contains cadherin-like domains in its extracellular portion. This multidomain extracellular module contains a binding site for a family of five related hetero-dimeric ligands. Each hetero-dimer is comprised of a secreted glial-cell line derived neurotrophic factor (GDNF) family ligand (GFL) and a membrane-anchored co-receptor GFRα (GDNF family receptor alpha). Once a GFL-GFRα ligand is bound to RET, this stimulates the activation of the receptor through tyrosine-based auto-phosphorylation. This mini-review explores how the shape and architecture of RET encodes a flexible GFL-GFRα binding site, summarising recent progress in understanding RET structure. It then discusses current views on how distinct assembles of GFL-GFRα-RET receptor complexes are able to activate the intrinsic RET tyrosine kinase function to relay intracellular signals.

## RET receptor tyrosine kinase architecture – function follows form

Receptor tyrosine kinases (RTKs) recognise a broad set of secreted ligand cues through a shared architecture comprising a unique multidomain extracellular module for ligand recognition coupled to a conserved intracellular kinase domain by a single-pass transmembrane helical segment [1]. This diversity in the extracellular module allows the 58 known human RTKs to recognize a wide variety of protein ligands to initiate specific cellular signalling responses [1]. The RET RTK is assigned to a single member subfamily due to the presence of multiple cadherin-like domains within its extracellular module (Figure 1A). These cadherin-like domains have diverged in sequence and structure, losing the adhesion function associated with canonical cadherin domains [2]. Instead, they encode a binding site for a GDNF family receptor alpha (GFRα) while an adjacent a cystine-rich domain (CRD) engages a glial-cell line derived neurotrophic factor (GDNF) family ligand. Unusually for RTKs, RET lacks paralogues (genes related by duplication within a genome) but instead, evolutionary pressure has expanded the number of ligands and co-receptors coinciding with the evolution of the neural crest in vertebrates [3, 4]. RET is known to respond to the five GDNF family ligands (GFLs): GDNF, neurturin (NRTN), artemin (ARTN), persephin (PSPN) and GDF15, when presented with their preferred GFL co-receptor to give GDNF-GFRα1, NRTN-GFRα2, ARTN-GFRα3, PSPN-GFRα4 and GDF15-GFRAL heterodimers [4]. A likely consequence of this ligand expansion is a broader repertoire of ligand signals, more responsive tissues and the acquisition of new ligand-co-receptor functions, some independent of RET signalling [5, 6]. An important question we address in this mini-review is: How is a single RET receptor able to recognise and accommodate each of the GFL family ligands when presented by their individual canonical co-receptors? To discuss this issue, we first describe the overall architecture of RET and the organisation of its three main structural components, the ligand-binding extracellular module (ECM), a single transmembrane helix (TM) that anchors RET in the plasma membrane, and an intracellular module (ICM) containing the intrinsic tyrosine kinase domain (TKD).

The RET ECM comprises a signal sequence, four cadherin-like domains (CLD1-CLD2-CLD3-CLD4), a cysteine-rich domain (CRD), followed by a short flexible extracellular juxtamembrane (eJM) segment (Figure 1A). Until recently, visualising the precise organisation of these domains been hampered by both the flexibility and the extensive glycosylation of the RET extracellular region. Crystallographic and cryo-electron microscopy analysis of the RET ECM have revealed its striking curvature and overall “C”-shaped domain organisation [7–10], with regions of localised flexibility (Figure 1B). These features arise from the shape of the individual CLD and CRD domains, their interdomain interfaces and the presence of multiple N-linked glycosylation sites. CLD1 is the most divergent region of RET across species in overall sequence conservation [11]. Structural evidence for this divergence is supported by a swapped disulphide between human and zebrafish CLD1 domains, with even more striking differences in disulphide patterns found in the insect clade RET orthologue [12]. The loss of calcium-ion coordinating residues between CLD1 and CLD2 is consistent with their folded clamshell domain arrangement and absence of calcium ions [12]. The limited interface between CLD2 and CLD3 retains the canonical cadherin triplet of calcium ions and coordinating acidic sidechains and is highly flexible [13]. In contrast, the hydrophobic interface between the heavily glycosylated CLD3 and highly basic CLD4 is calcium-free and gives the RET ECM its curved shape [7, 10]. The CRD extends from the end of CLD4 up to residue 634 (human RET numbering) and is comprised of two distinct regions. The first part forms a rigid globular domain containing five disulphide bridges and an EF-hand motif that binds a single calcium ion and packs against CLD4 [7, 10]. The second part is a flexible unstructured region known as the extracellular juxtamembrane (eJM) that contains a further three disulphide bridges. These eJM cysteine residues are important sites targeted by oncogenic mutation in the endocrine cancer MEN2A, most frequently at C630 and C634 [14].

Residues 635 to 657 of human RET are predicted to form a transmembrane helix (RET-TM) with similar length to those observed for other RTKs [15, 16]. The membrane-spanning TM is predominantly hydrophobic, apart from three polar serine residues that contribute to signalling [17]. RET-TM homodimerization has been demonstrated and is essential for oncogenic activation [17]. At the end of the RET-TM is a cysteine motif C-X-X-C resembling an S-palmitoylation site also found in CD4 [18], hinting at a role in controling RET localisation and downstream signaling [19].

The RET intracellular portion contains a 66-residue long juxtamembrane (iJM) prior to the TKD (Figure 1A). It also extends beyond the TKD into a carboxyl-terminal tail that differs between the RET9 and RET51 splice isoforms (see Figure legend) [14]. The iJM and tail regions flanking the TKD appear to be flexible, and accordingly have not yet been observed in crystal structures. Both have roles in autoinhibition of the inactive receptor and stabilisation of an active kinase conformation [20, 21]. The extremities of the ICM contain important sites of tyrosine phosphorylation that engage binding partners for downstream signalling. The iJM contains Y687 which is targeted by autophosphorylation to create a binding site for SHP2 [22]. It also has a protein kinase A phosphorylation site at S696 which can also signal, but may suppress the neighbouring Y687 phosphorylation [23].

Following the iJM is the critical TKD catalytic core, with the shared bilobal architecture of eukaryotic protein kinases to generate a nucleotide ATP-binding site and a substrate-binding site used for either cis- or trans autophosphorylation [24, 25]. In analyses of kinome phylogeny, the RET TKD is most similar to that of the FPVR kinases (fibroblast, platelet-derived, and vascular growth factor receptors) [26]. Nucleotide-bound structures of the RET TKD have been determined for its “active” autophosphorylated state (DFG-motif in) (Figure 1B), with aligned catalytic and regulatory spines similar to those of many other active kinase conformations [27]. The canonical RTK activation loop in RET harbours two tyrosine residue at 900 and 905 that are phosphorylated upon RET activation [28]. These sites are proposed to engage Grb7/Grb10 when phosphorylated [29, 30]. Absent is third cis-inhibitory tyrosine found in the activation loop of many other RTKs [31]. Kinetic studies on recombinant RET kinase domain suggests the unphosphorylated form of RET exhibits catalytic activity comparable to the phosphorylated form with an almost identical conformation [27]. While a nucleotide-free and/or autoinhibited state has not yet been described for RET TKD, the exact nature of the RET-TKD regulatory mechanism is not yet clear which needs addressing.

After the RET-TKD, an unstructured “C-terminal tail” segment contains autophosphorylation sites for recruiting PLC-gamma (Y1015) and a cis-autophosphorylation at Y1062 site. Y1062 is the key multi-protein docking site on RET required for biological activity as well as transforming activity of its oncogenic forms [28]. Multiple partners assembled onto this site include SHC, FRS2, Enigma, DOKs and IRS1/2. Partners such as the lipidated-FRS2 PTB adaptor and the non-lipidated-SHC PTB adaptor influence the composition of RET signalling assemblies and which lipid compartment they are recruited to [32–34]. Finally, the two main RET isoforms known as RET9 and RET51 have different C-terminal sequences beyond glycine-1063, with the shorter RET9 isoform ending at 1072 and RET51 extending to 1114. RET51 contains the splice form-specific Y1090 and Y1096 autophosphorylation sites [35]. The latter Y1096 is able to recruit Grb2, enabling coupling to a sustained RAS–ERK signaling [36].

### Encoding a flexible GFL-GFRα binding site

Each GFL adopts a cystine-knot [37] and forms a covalent homodimer with a dimerization mode similar to TGF-ß family ligands [38]. The GFL co-receptors have three related helical-rich domains D1-D2-D3 (except for GFRα4) that are organised topologically as D1-D3-D2 with long connecting linkers (Figure 1C). In each case the tips of GFL ß-strand “fingers” engage domain D2 of their corresponding GFRα co-receptor to give a 2:2 complex with a “U”-shaped architecture, where each GFRα subunit forms an arm of the “U” tethered by the bivalent GFL ligand (Figure 1C). Differences in the angle between the “arms” formed by the GFRα in the 2:2 complex are evident between the different structures determined [39, 40].

How does the RET architecture accommodate each ligand-co-receptor pair? For each GFL, residues from each GFL protomer of the dimer form a concave surface complementary to the convex shape of the RET CRD domain [9]. This interaction broadly resembles the contacts made by many TGF-ß ligands to engage their receptors [38]. However, for each GFL these contacts alone are not sufficient to form a stable RET interaction but require their membrane-anchored co-receptor [41, 42]. Recent structures of different GFL-GFRα complexes bound to RET-ECM revealed a direct role for the GFRα subunits in engaging RET [40, 43–45]. Each GFRα binds adjacent to the small flexible CLD2-CLD3 calcium-ion interface through a GFRα D3 domain contact, involving a conserved CX_4_N/QX_1-2_EEX_0-2_C helical-turn motif. Comparison of ligand-bound and ligand-free RET-ECM structures have revealed conformational changes required to clamp onto a GFRα subunit, pivoting about the limited CLD2-CLD3 interface [7]. Recognition of GFRα-specific elements also play a role, for example the most divergent GFRAL makes unique contacts to CLD1, CLD2 and CLD3, revealing a conformational adaption [7]. The conclusion is that interdomain plasticity within RET-ECM assists with the flexible recognition of the divergent GFRα family members (Figure 1C).

How are RET-ECM arranged through these spatially separated and independent GFL and GFRα contacts [7–10]? Recruitment of two “C”-shaped RET subunits to form a 2:2:2 ternary complex generates an assembly architecture that has been described as a figure-of-eight (when viewed from above) and as GFRα-RET “batwings” (viewed from the side) [8–10]. The angle formed between the RET-GFRα batwings varies substantially between different GFL-GFRα-RET complexes with GDNF-GFRα1 and GDF15-GFRAL showing the widest and narrowest extents respectively (Figure 1C). However, it is not yet clear whether these differences in receptor-ligand complex geometry reflect functionally different signalling outputs. A surprise finding from structural studies was that the spatial separation of the RET dimers observed in 2:2:2 assemblies formed with different GFL-GFRα pairs is almost exactly conserved across both GFL-GFRα paralogs and clades (Figure 1C). This suggests that the precise inter-RET spacing imposed by hetero-dimeric ligand binding despite adaptions, is a conserved property which is important for receptor activation and signalling.

The GFL-GFRα-RET complex architecture also explains a conundrum whereby no single domain within the RET ECM was found to be sufficient to bind GFL-GFRα ligands. Instead, the discontinuous nature of the GFL-GFRα binding epitope requires the entire RET ECM [9]. A contributing factor is the folding dependencies for CLDs. For example, the CLD1-2 clamshell and buried surface are required for this portion to fold as a single globular unit, whilst the CLD3 contains most of the calcium-coordinating ligands. CLD4 shares a substantial interface with CRD that is in turn presented to GDNF, forming crucial contacts with both GDNF protomers. Therefore, the CLD1-CLD4 and CRD organisation within RET conveniently explains why all domains are required both for proper RET folding and ligand-co-receptor recognition.

### From ligand engagement to receptor activation and beyond

How then does recognition of hetero-dimeric GFL-GFRα ligands by RET stimulate its activation and downstream signalling? Likely contributing factors include: ligand-driven allosteric changes, ligand-binding kinetics, the activated RET receptor lifetime, overcoming auto-inhibitory regulation and receptor dimerization/multimerization state(s). Some of these properties have been defined in detail and others have not been addressed at all. To date, the different RET domains characterised (CLD1-CLD2), ECM, TM and TKD) have all been shown to form dimers by a variety of methods [10, 12, 17, 27]. This implicates RET dimerization as being central to signalling. Current evidence for the unliganded state of RET supports a pre-formed RET dimer mediated through a CLD1-CLD2 interface that has been observed both in a crystal structure and inferred from cryo-EM of soluble RET ECM dimers [10, 12]. This proposed ground state of RET dimers could potentially spatially separate both TKDs preventing spurious activation, analogous to the mechanism proposed for the IGFR structure [46]. In such a scenario, an allosteric activation mechanism triggered upon hetero-dimeric GFL-GFRα ligand binding would disrupt the CLD1-CLD2 dimer by binding at the CLD2-CLD3 junction (Figure 1E). This could then reposition each RET transmembrane segment with their high affinity for self-association, to adopt an active dimer configuration aligning both TKDs for *trans*-autophosphorylation. For a robust regulatory mechanism to operate it would either need to prevent RET-TM dimerisation in the absence of ligand or to capture a signalling “inactive” dimeric TM arrangement.

The impact of RET-TM dimerisation on the intrinsically flexible iJM and tail regions of RET, harbouring key auto-phosphorylation site tyrosines is unclear (Figure 1D). If the ECM and ICM portions are conformationally coupled by the RET-TM after ligand-binding, the iJM and tail regions could become rapidly accessible and phosphorylated. However, the determination of a full-length RET structure to address this issue has not yet been reported. Cryo-EM imaging from many labs on different RTKs have consistently failed to see coupling of ECM and ICM, in all cases resulting in well ordered ECM structures but only low resolution ICM regions [47–49]. A likely explanation is that they are flexibly linked and that enforced proximity of TKDs arising from ligand dimerisation may be sufficient for activation. This remains a plausible scenario for RET activation as well.

Structural studies on RTK TKD domains have shown many different dimerization modes unique to individual RTKs from obligate trans-dimers to allosteric asymmetric dimers [50, 51]. Most crystal forms of isolated RET TKD adopt a head-to-tail inhibited dimer with the substrate pocket inaccessible [27]. To us this suggests the precise arrangement of an activated RET TKD dimer has not yet been captured. Studies on recombinant RET ICM *in vitro* have provided evidence for a two-state model for the activation of the TKD [21]. This process involves *cis*-phosphorylation of Y687 (iJM) and Y1062 (tail) which flank the TKD which are rapidly targeted and constitute “early” sites (Figure 1D), Whether phosphorylation of the early *cis*-sites leads to stabilisation of an active state, or overcoming autoinhibitory elements, or both, is not yet clear. Subsequently, the slower *trans*-phosphorylation of sites at Y900/Y905 situated in the activation loop crucial for RET signalling accumulate. An investigation of RET autophosphorylation kinetics in a cellular context supported a more synchronized mode of tyrosine phosphorylation [52]. Further validation is needed to reconcile these in vitro and in cellulo findings, requiring better antibody tools to monitor more precisely the kinetics of full length RET activation in a cellular membrane. *In vitro* analysis of RET phosphorylation trajectory by removing individual sites by Y>F mutation did not impact the phosphorylation of other tyrosine sites [21], suggesting no precise ordering of tyrosine sites in RET but different phosphorylation kinetics for each site. This contrasted studies on the closely related RTK FGFR, where autophosphorylation of tyrosine residues has been shown to be sequentially ordered in time, each serving as docking sites for downstream signalling proteins [41].

RTKs are thought to continuously cycle between active and inactive states, as evidenced by the rapid impact of TKI inhibitors on phosphorylation site lifetimes [53]. This constant ATP-dependent recycling together with the need for multi-site phosphorylation and the persistent action of phosphatases may act as an error filter to discriminate genuine activating signals from noise. A time lag between initial receptor-ligand interaction and the formation of active, phosphorylated complexes and consequently further recruitment of downstream signal transducers may help in this regard (Figure 1E). The different GFL-GFRα complexes are likely have slightly different on and off rates for engaging RET and similar but distinct conformations [7, 10]. Whether such differences influence the conformation and persistence of active RET receptor remains to be shown.

Many outstanding questions remain that limit our understanding of RET signalling. Evidence for the auto-inhibitory mechanism of RET is still circumstantial. Beyond a 2:2:2 stoichiometric complex of GFL-GFRα-RET reported, independent groups have observed different 4:4:4 assemblies for a NRTN/GFRα2/RET complex, a MEN2A pathological variant of RET and zebrafish GDNF-GFRα1-RET [7, 10, 54]. Are these multimeric assemblies relevant to physiological RET signalling or pathophysiological contexts? Is there a role for proteoglycan binding in RET signalling by GDNF, in view of the published heparan sulfate binding site within GDNF [55]? Are there different signalling outputs and phosphotyrosine-binding effector complexes assembled for different GFL-GFRα pairs given their different ligand-RET receptor geometries? Tools and technologies to address these questions are now available indicating an exciting future ahead for RET signalling mechanisms.

It is instructive to consider how current insights can inform on the design of better drugs targeting RET-driven cancers and preventing drug resistance arising? Next-generation ATP-competitive inhibitors of RET and combinations are still being developed to tackle known resistance mutations and bypass mechanisms [56]. For other kinase targets, developing allosteric inhibitors as an orthogonal modality to ATP competitive inhibitors has been successful as a route to alleviate kinase drug resistance [57]. Another promising approach is targeted protein degradation by PROTACS through hijacking ubiquitin-proteasome/lysosomal pathways to tag and destroy disease-causing RET variants [58]. Equally, biologics targeting the extracellular portion of RET may provide an alternative strategy to antagonise RET activation either alone or as antibody drug conjugates. Finally, strategies to develop peptide antagonists to specific GDNF-GFRα pairs are progressing [59]. The broader picture indicates that clinicians treating RET-driven disease still urgently need better treatments but there is optimism among scientists driving forward innovative ideas to deliver them.

## Conclusions

In this mini-review we have described progress in determining RET receptor architecture, revealing how it can bind and flexibly accommodate a family of five ligands when presented by membrane-linked co-receptors. The co-receptors themselves are now known to be a central part of the hetero-dimeric ligand by directly binding to RET. Bivalent heterodimeric ligand complexes recruit two RET receptors with distinct geometries but almost identical separation, a feature likely crucial for receptor activation. Plasticity in RET-ECD allows the accommodation of all five GFL-GFRα ligands with unique adaptations. Current models for RET activation favour a shift from an autoinhibited basal state in which RET is dimeric, to a clamped GDNF-GFRα-RET ternary complex, though higher order assemblies may also be relevant. For signal transduction to progress, receptor occupancy by the heterodimeric ligand likely permits transmembrane segment dimerisation thereby enforcing the close proximity of the TKD from each protomer. This may be sufficient to stimulate the formation of cis- and trans-autophosphorylation sites triggering a persistant activated RET conformation able to assemble a phospho-tyrosine-based multi-protein signalling hub. Structural and mechanistic insights described here are enabling new approaches to drugging RET, potentially expanding the repertoire of molecules and biologics available for treating RET-driven disease.

## Figures and Tables

**Figure 1:** (A) Schematic of human RET sequence highlighting modules, individual domains, calcium-binding sites, auto-phosphorylation sites and their downstream effectors and corresponding residue numberings. The two abundant RET isoforms RET9 and RET 51 extend to residue 1072 or to 1114 respectively. RET51 is unique in containing the Y1096 site for binding to Grb2. (B) Overview of the three-dimensional structure of the human RET ECM (left panel), with domain colours coded according to panel (A), indicating the location of binding sites, and the human RET ICM in the unphosphorylated state (right panel). The RET ECM structure is a predicted model using AlphaFold3 [60] and the RET ICM model is PDB accession 2IVT. (C) Modular domain structure of GFRα1 and GFRAL and a schematic for GFL indicating their dimeric nature. Orthogonal views of schematized views of GDNF-GFRα1 and GDF15-GFRAL assemblies with RET ECM. Images are derived from published structures [7, 10]. The similar spacings close to the membrane of both RET protomers is highlighted as well as the plasticity evidenced between the structures of RET with different GFRα-GFL pairs, notably the D1 domain positioning. (D) Schematic of RET ICM before and after ligand-induced activation, emphasising the 2-step mechanism proposed involving rapid and slow auto-phosphorylation sites shown in vitro and the opening up of an autoinhibited RET ICM conformation. (E) Proposed functional states for RET assemblies highlighting an inactive dimeric state, a speculative RET ECM complex with GFRα1, an active 2:2:2 assembly and a proposed higher order 4:4:4 multimer of GDNF-GFRα1 and RET.
